# Artificial Intelligence-based Machine English-Assisted Translation in the Internet of Things Environment

**DOI:** 10.1155/2022/7428563

**Published:** 2022-08-05

**Authors:** Wanfang Zhang, Yuan Tang

**Affiliations:** ^1^School of Foreign Languages, Wuhan Polytechnic University, Wuhan 430023, Hubei, China; ^2^School of Humanities and Arts, Jiaxing Nanhu University, Jiaxing 314000, Zhejiang, China

## Abstract

With the development of Internet of Things technology, the things that machines do instead of humans are becoming more and more complicated. Machine translation has developed rapidly in the past few decades, and the translation system has also been greatly improved. People's life and work are inseparable from machine translation, which brings a lot of convenience to people. But machine translation also has many flaws. Although machine translation can translate long texts in a very short time, its translation quality is quite poor, especially in the face of advanced English such as professional English, terminology, abbreviations, etc. To this end, machine English-assisted translation systems have been developed in recent years. Different from the working principle of machine English translation, machine English-assisted translation is a method of artificial intelligence + human-computer interaction. It uses convolutional neural networks and deep learning to translate words efficiently. The translator puts the original text and the translation into the machine database each time, and the machine can process some English terms, complex sentences, technical English, and other advanced English after continuous learning. Machine English-assisted translation can reduce repeated translations and greatly improve translation quality and translation efficiency. In this paper, the combination of artificial intelligence and machine English-assisted translation is compared with machine English translation, and comparative experiments are carried out by setting different matching degrees. Experiments show that the translation efficiency of machine English-assisted translation is much better than that of machine English translation. As the matching rate increases, the translation efficiency of machine English-assisted translation is higher. When the matching rate is greater than 80%, the translation efficiency is three times that of machine English translation. However, it is slightly insufficient in processing pure, simple statements. It highlights the advantages of machine English-assisted translation in terms of term translation and long complex sentences.

## 1. Introduction

With the advance of time, technologies such as artificial intelligence and neural networks have had a huge impact on social production and life. People are gradually abandoning dictionaries to look up meanings in different languages. In the 1950s, IBM Corporation of the United States translated several simple foreign languages into English for the first time, and the world's first machine translation experiment was successful. Machine translation has also entered people's lives from now on. With the development of machine translation today, from the initial translation of dozens of words at a time to the translation of the entire article, it has now become a huge translation system. The benefits of machine translation are self-evident, but there are also many disadvantages. It cannot deal with technical English, English terminology, complex sentences, and other sentences that need to be translated by people. Machine translation is simply literal translation. A new translation system has developed rapidly in recent years. Machine English-assisted translation is a translation mode of human-computer interaction. Its translation memory technology can efficiently handle a large number of repeated sentences and can translate complex English that cannot be translated by machine English. English is an international language, and people communicate through English in many cases. The combination of machine English-assisted translation and artificial intelligence technology solves many defects in ordinary machine English translation and greatly improves translation efficiency and quality.

This paper focuses on the topic of machine English-assisted translation based on artificial intelligence. This paper has the following innovations: (1) It sets different match rates (all characters of a segment + the percentage of characters in the format of the translation memory content), experimenting with comparing the efficiency and quality of machine English-assisted translation and machine-English-assisted translation. (2) The advantages of machine English-assisted translation in the translation of complex English fields such as technical English and terminology are proved through experiments. Therefore, this study is innovative.

## 2. Related Work

With the development of Internet of Things technology and artificial intelligence, human-computer interaction technology is combined with many fields. In order to improve the quality and efficiency of translation, more and more people are investing in machine translation. Among them, the Li and Chen study evaluated four aspects of machine translation. Machine translation still has many defects and cannot completely replace human translation [1]. Castilho et al. compared neural machine translation with ordinary machine translation through experimental research and found that machine translation based on a neural network is faster in translation efficiency [2]. Miura et al. learned through experiments that statistical-based machine translation has high translation accuracy [3]. However, the methods used for machine translation are too inefficient and not accurate enough.

In recent years, with the development of deep learning technology, machine English-assisted translation has gradually entered the field of vision. Among them, Alarifi and Alwadain studied a statistical-based machine English-assisted translation system, using techniques such as machine learning to process English phrases [4]. Saleh Mahdy Mohammed et al. studied translators' skills in using machine English-assisted translation by means of a questionnaire. Studies have shown that the use of machine English-assisted translation can greatly improve translation efficiency [5]. The Vandenberg study aimed to illustrate that Artificial Intelligence-based machine-assisted translation takes less time and effort than human translation [6]. Balashov research pointed out that artificial intelligence technology plays a crucial role in the study of machine-assisted translation and machine translation [7]. Fu research showed that machine English-assisted translation can help improve English learning [8]. Through the inspiration and experimental conclusions of other researchers, the shortcomings of machine English translation are known, and it is determined that the research of machine English-assisted translation based on artificial intelligence is feasible. Its disadvantage is that the translation efficiency is not as good as machine translation when translating short and simple sentences. Machine English-assisted translation requires a lot of training to perfect its self-learning process.

## 3. Artificial Intelligence-Based Machine English-Assisted Translation Method

### 3.1. Neural Network Technology

Artificial neural networks are based on the way the human brain processes information. The complex computing process of the neural network is processed by extracting neurons as nodes [9, 10]. With the development of time, scientists have perfected the theory of neural network technology, and neural network models of various structures have been proposed one after another [11]. From the original BP neural network to the Boltzmann machine, convolutional neural network, etc., neural network technology has a very mature concept in the study of intelligent mechanisms [12–14]. At present, neural network technology has been applied to various fields of intelligent computing, which has brought great convenience to people.

#### 3.1.1. BP Neural Network

The structure of BP neural network is divided into three layers: input layer, hidden layer, and output layer. The structure diagram of the BP neural network is shown in Figure 1. It can be seen from the structure diagram of the BP neural network that any input value can map an output value, and the self-learning of the neural network can be realized by training a large amount of data [15].

The algorithm principle of the BP neural network is that the input layer receives the stimulus. That is, it receives the data information and then transmits the data to the hidden layer. After receiving the data, the hidden layer processes the data through the connection weights and activation functions between the neuron nodes and then passes it to the output layer. The output layer compares the actual result with the expected result by sorting out the data information passed from the hidden layer. If the difference between the actual result and the expected result is not within an acceptable range, the information is passed backward. That is, from the output layer to the hidden layer and then to the input layer, by modifying the weights of neurons, the loop is ended until the difference between the actual result outputted by the output layer and the expected result is within an acceptable range, and the process of self-learning is achieved.

The BP neural network algorithm is divided into two processes: forward propagation and backpropagation [16]. The forward propagation path data goes from the input layer-hidden layer-output layer. The processing state of neurons in each layer affects the neurons in the next layer. If the actual output of the output layer is very different from the expected output, then there will be a backpropagation of the error. That is, the error will go from the output layer-hidden layer-input layer. The two ways of propagation make the actual output infinitely close to the expected output.

*(1) Forward Transfer Process.* It takes the three-layer structure of the BP neural network as an example and sets the input layer nodes as *a*, the hidden layer nodes as *b*, and the output layer nodes as *c*. The weight of the connection between the input layer and the hidden layer is *w*_*ij*_. The node threshold of the hidden layer is represented by *b*_*i*_, and the weight of the connection from the hidden layer to the output layer is *w*_*jk*_. The node threshold of the output layer is denoted by *d*_*j*_ [17]. The connections between neurons in the BP neural network structure are very complex. The calculation of the BP neural network also relies on the sum operation of the output value and the weight value of each time element.

So the output of the hidden layer is expressed as follows:

(1) $$\begin{array}{c} Z_{i}=f\left(\sum_{j=1}^{a}w_{ij}x_{j}+b_{i}\right). \end{array}$$

Similarly, the output of the output layer is expressed as follows:

(2) $$\begin{array}{c} S_{j}=f\left(\sum_{k=1}^{b}w_{jk}Z_{j}+d_{j}\right). \end{array}$$

In formulas (1) and (2), the function *f*() is the activation function, *i*, *j*, and *k* are the nodes corresponding to each layer.

*(2) Reverse Transfer Process*. The main working principle of the BP neural network is the reverse transmission of the error, and then the weights and thresholds of the neurons are changed so as to achieve the self-learning purpose of the BP neural network. If the input layer has *g* sample input, then when the *v*^th^ sample is input, the output result obtained by the overall network is *y*_*j*_^*v*^. Among them, *v*=1,2,…, *g*, *j*=1,2,…, *b*. It calculates the squared error of the sample at this time and can get the following:

(3) $$\begin{array}{c} E_{v}=\frac{1}{2}\sum_{j=1}^{b}{\left(t_{j}^{v}-y_{j}^{v}\right)}^{2}. \end{array}$$

In formula (3), *t*_*j*_^*v*^ is the expected output.

Performing error analysis on *g* samples, the average error formula can be obtained as follows:

(4) $$\begin{array}{c} E=\frac{1}{2}\sum_{v=1}^{g}\sum_{j=1}^{b}{\left(t_{j}^{v}-y_{j}^{v}\right)}^{2}=\sum_{v=1}^{g}E_{v}. \end{array}$$

By expressing the change of the weight Δ*w*_*jk*_ of the output layer, it can get the following:

(5) $$\begin{array}{c} \Delta w_{jk}=-\eta \frac{\partial E}{\partial w_{jk}}=\sum_{v=1}^{g}\left(-\eta \frac{\partial E_{v}}{\partial w_{jk}}\right). \end{array}$$

In formula (5), *η* represents the learning efficiency.

Then the signal formula of the error is expressed as follows:

(6) $$\begin{array}{c} \sigma_{yj}=-\frac{\partial E_{v}}{\partial S_{j}}=-\frac{\partial E_{v}}{\partial y_{j}}\cdot \frac{\partial y_{j}}{\partial S_{j}}. \end{array}$$

It transforms formula (6) to get the following:

(7) $$\begin{array}{c} \sigma_{yj}=\sum_{j=1}^{b}\left(t_{j}^{v}-y_{j}^{v}\right)f^{\prime }\left(S_{j}\right). \end{array}$$

In formula (7), *f*′(*S*_*j*_) is the derivative of *S*_*j*_

By changing the formulas (5) and (7), the weight change formula between neurons in the output layer can be obtained as follows:

(8) $$\begin{array}{c} \Delta w_{jk}=\sum_{v=1}^{g}\sum_{j=1}^{b}\eta \left(t_{j}^{v}-y_{j}^{v}\right)f^{\prime }\left(S_{j}\right)\cdot Z_{i}. \end{array}$$

Then the weight change formula between each neuron in the hidden layer is as follows:

(9) $$\begin{array}{c} \Delta v_{ij}=\sum_{v=1}^{g}\sum_{j=1}^{b}\eta \left(t_{j}^{v}-y_{j}^{v}\right)f^{\prime }\left(S_{j}\right)w_{jk}f^{\prime }\left(S_{i}\right). \end{array}$$

BP neural network has a strong input-output mapping relationship and is often used in machine recognition, data mining, data classification, text translation, and other fields. However, when the input of the BP neural network increases, the time and space it takes to train will also increase, making the training result very slow.

#### 3.1.2. Convolutional Neural Network

Since artificial neural networks have many drawbacks in data processing, a large amount of data is required for training. Once the amount of data reaches the threshold, the processing mechanism of the network system becomes very slow. In order to change the drawbacks of artificial neural networks, relevant scholars have changed the three-layer structure of artificial neural networks to an end-to-end data structure. This structure is very suitable for text translation, thereby reducing the training data and improving the processing efficiency of the neural network. A new neural network model is formed through the transformation of the BP neural network. A convolutional neural network is a neural network algorithm that includes a convolution algorithm and has deep learning capabilities [18–20]. The structure of a convolutional neural network mainly includes a convolutional layer, subsampling layer, and fully connected layer [21]. The structure diagram of the convolutional neural network is shown in Figure 2.

*(1) Convolutional Layer*. The main task of the convolutional layer is to perform feature extraction. The main features of this layer are local sensitivity, shared parameters, and multiple convolution kernels. Local sensitivity originates from the stress response of biological nerves to external stimuli. When neurons are farther apart, their sensitivity decreases. When neurons are closer together, their sensitivity increases. To reduce the complexity of the network, each neuron in the convolutional layer only senses changes in the surroundings. The extraction of omnidirectional feature vectors is generally performed by adding convolution kernels [22].

*(2) Subsampling Layer*. Subsampling layers are also known as pooling layers. The main purpose of the subsampling layer is to perform statistics on the feature vector output by the convolutional layer. The network dimension can be reduced as much as possible after the pooling operation of the feature vector, and the weight parameters of the neuron nodes can be reduced [23]. There are three sampling rules for the subsampling layer: equal sampling, peak sampling, and random sampling. Mean sampling is the sample collected after averaging each area. Peak sampling is to select the largest value in each area as the sampling sample. Random sampling is to randomly select the value of each area as a collection sample.  Figure 3 is a sampling diagram of the subsampling layer.

*(3) Fully Connected Layer*. A fully connected layer means that neurons are completely connected to the input data. The fully connected layer plays a classification role in the entire convolutional neural network.

### 3.2. Translation Memory Technology

“Translation Memories” (TM) is the core function of machine-assisted translation. A translation memory is formed by storing the translated sentences and the corresponding original texts in a database. When translating sentences later, the system will automatically search for the same sentence as the translation memory to avoid repeated translations. This greatly improves the speed and efficiency of translation. The core technology of translation memory is to quickly find sentences in translation memory through deep learning technology and express their corresponding translations [24].

Deep learning is a brand new approach in the field of machine learning. The research model is derived from an artificial neural network [25, 26]. Deep learning processes data such as pictures, sounds, and text information, imitating the brain's processing of information. It extracts feature vectors hierarchically from the training data and passes the extracted features to the next layer hierarchically. This makes the information obtained by the later neurons more specific. This kind of training is very suitable for the translation of text. Typical deep learning algorithms are deep belief networks and deep Boltzmann machines.

#### 3.2.1. Deep Belief Network

Deep belief network is a probabilistic model network structure. Compared to BP neural network, the deep belief network model can observe the connection between data and labels. Deep belief networks can evaluate both prior and posterior probabilities. But BP neural network can only evaluate the posterior probability, so the deep belief network structure makes up for many shortcomings of the BP neural network. For example, BP neural network requires a large number of samples for training. The learning process of the traditional feedback neural network is very slow, and the error needs to be fed back layer by layer. The loop algorithm finally obtains the desired output, and it is difficult to achieve global optimization. If it is used in translation, the translation efficiency will be very slow. Usually, in BP neural network, the selection of samples is very important. Once the sample selection has a large deviation, the local optimum of the result will appear instead of the global optimum [27]. The deep belief network structure is shown in Figure 4.

The deep belief network structure is a three-layer structure. Its basic processing node is a restricted Boltzmann machine. Neurons between layers are connected in a bidirectional or unidirectional manner. Neurons between the same layers cannot communicate. The top layer is a directionless restricted Boltzmann machine. The other limiting Bozeman machines are all top-down delivery.

#### 3.2.2. Deep Bozeman Machine

A deep Boltzmann machine is a symmetric and multilayered neuron structure. Its neuron nodes consist of random 0s or 1s. A deep Boltzmann machine has an input layer. It sets its neuron unit as *V*, then *V* ∈ {0,1}. The network structure has multiple hidden layers at the same time. It sets the neural units of the hidden layer as *x*_1_, *x*_2_, *x*_3_, then *x*_1_, *x*_2_, *x*_3_ ∈ {0,1}. In this neural network, neuron nodes in adjacent layers are connected to each other. Neuron nodes in the same layer are not connected. The weight matrix of the input layer and any hidden layer is a parameter denoted by *W*. Deep Boltzmann machines are represented by a series of parameters [28]. The structure of the deep Bozeman machine is shown in Figure 5.

In Figure 5, *W*_1_ is the weight matrix of *V* and *x*_1_, and then the energy of the deep Boltzmann machine is expressed as follows:

(10) $$\begin{array}{c} E\left(V,x,W\right)=-V^{T}W_{1}x_{1}-x_{1}W_{2}x_{2}-x_{2}W_{3}x_{3}. \end{array}$$

In formula (10), *E* represents the entire deep Boltzmann machine energy. *T* is the transposition of the matrix.

The neuron probability function of the input layer is as follows:

(11) $$\begin{array}{c} P\left(V,W\right)=\frac{1}{Y\left(W\right)}\sum_{x}\exp\left(-E\left(V,x_{1},x_{2},x_{3}\right)\right). \end{array}$$

In formula (11), *Y*(*W*) is the analysis function. Exp is an exponential function with the base *e* of the natural constant, and its mathematical expression is as follows:

(12) $$\begin{array}{c} Y\left(W\right)=\sum_{v}\sum_{x}\exp\left(-E,x_{1},x_{2},x_{3}\right). \end{array}$$

The distribution of the input layer and hidden layer is as follows:

(13) $$\begin{array}{c} P\left(x_{1}^{j}=1|V,x_{2}\right)=\sigma \left(\sum_{j}W_{1}^{ij}V^{i}+\sum_{k}W_{2}^{kj}x_{2}\right), \end{array}$$

(14) $$\begin{array}{c} P\left(x_{2}^{k}=1|x_{1},x_{3}\right)=\sigma \left(\sum_{j}W_{1}^{jk}x_{1}^{j}+\sum_{m}W_{3}^{km}x_{3}^{m}\right), \end{array}$$

(15) $$\begin{array}{c} P\left(x_{3}^{m}|x_{2}\right)=\sigma \left(\sum_{k}W_{3}^{km}x_{2}^{k}\right), \end{array}$$

(16) $$\begin{array}{c} P\left(V_{i}|x_{1}\right)=\sigma \left(\sum_{j}W_{1}^{ij}x_{1}^{j}\right). \end{array}$$

Formulas (13)–(16) can jointly calculate the probability distribution of each layer of the input layer and the hidden layer, where it is a logistic function.

(17) $$\begin{array}{c} \sigma \left(x\right)=\frac{1}{1+e^{-\left(x\right)}}. \end{array}$$

#### 3.2.3. Restricted Boltzmann Machine for Layer-by-Layer Training

A restricted Boltzmann machine is an unsupervised neural network model. It is an improved version of the deep Bozeman machine. After learning the deep Boltzmann machine layer by layer, the parameters of each layer are adjusted to make the network learning move in the expected direction.

After learning the first layer of the deep Boltzmann machine, its corresponding distribution probability is as follows:

(18) $$\begin{array}{c} P\left(V,W\right)=\sum_{x_{1}}P\left(x_{1},W_{1}\right)P\left(V|x_{1},W_{1}\right). \end{array}$$

After learning the second layer, if the distribution probability of the second layer is better than the first layer, replace the probability of the first layer with the probability of the second layer. Similarly, when the probability of the third layer is better than that of the second layer, the probability of the second layer can be replaced by the probability of the third layer so that the entire network model can be optimized.

### 3.3. Human-Computer Interaction Technology

Machine-assisted translation is a process of human-computer interaction. People save the original text and the translation into the machine. After the machine recognizes it, it regularly recognizes the later translated text and then presents it to people for them to choose. As the number of recognitions increases, so does the translation accuracy. An interactive model based on positive feedback is used for this. It can select bilingual as positive feedback to limit the decoding of the translation system when translating [29].

#### 3.3.1. Prefix Human-Computer Interaction Translation

Prefix human-computer interaction translation is a traditional interaction method. It is mainly through the prefix to carry out a full-text search. The working process is as follows: let the translation source file be *k*, the translation prefix be *t*_*a*_, and the translation system predicts the most matching suffix of the translation according to the prefix and the source file:

(19) $$\begin{array}{c} t_{b}=\text{argmax}P_{u}\left(t\right)\cdot P_{v}\left(k|t\right). \end{array}$$

In formula (19), *t* is the full text of the translation, *t* is composed of *t*_*a*_ and *t*_*b*_, and argmax is a function of the set. *P*_*v*_(*k|t*) is the translation model, and *P*_*u*_(*t*) is the language type. The prefix-based human-computer interaction translation system calculates the suffix of the translation by using the translation model. The suffix files are filtered in combination with the translation and prefix matching. In this translation method, the prefix of the translation is used for retrieval and the suffix translation is screened accordingly, and the translation suffix resource is not used. For translation in this way, the suffix text of the translation cannot be saved, which may easily cause information loss.

#### 3.3.2. Fragmented Human-Computer Interaction Translation

In the fragmented human-computer interaction translation system, the use of the system's translation is not limited to the prefix but can save the correct fragment in the suffix translation. This method solves the shortcoming of the prefix-type human-computer interaction translation that cannot use suffix resources. The translation system will predict and translate sentences with incomplete suffixes. The formula is as follows:

(20) $$\begin{array}{c} h_{1}^{N}=\text{argmax}P\left(h_{1},\ldots ,h_{N}|k,f_{1},\ldots ,f_{N}\right). \end{array}$$

In formula (20), *h*_1_^*N*^=*h*_1_,…, *h*_*N*_ is the unidentified sequence fragment and *f*_1_, *f*_2_,…, *f*_*N*_ is the true fragment in the suffix.

The fragmented human-computer interaction translation mode also has obvious shortcomings. Fragments are mostly single words, which are difficult to align with sentences in the source file after translation. The system can only translate the following text based on the fragments connected behind the previously generated words and cannot guarantee the alignment of the source file and the translation.

#### 3.3.3. Positive Feedback Human-Computer Interaction Translation

The positive feedback human-computer interaction mode just solves the problem that the source files cannot be aligned with the translation fragments in the fragmented translation. This method is suitable for translated text [30]. In the positive feedback mode, the system will provide translation options for each segment, and the translator can also use the segment in the form 〈*f*_*i*_, *d*_*i*_〉 to translate. The formula is as follows:

(21) $$\begin{array}{c} t=\text{argmax}P\left(f_{1},d_{1},\ldots ,f_{N},d_{N},t|k\right). \end{array}$$

In formula (21), *d*_*i*_ is the translation of the corresponding source file *f*_*i*_.

## 4. Experiment of Machine English-Assisted Translation Based on Artificial Intelligence

### 4.1. Experiments on the Validity of Translation Samples

#### 4.1.1. Sample Data

In order to make an all-round comparison between the two translation modes of machine English-assisted translation and machine English translation, the samples selected for the experiment must be strictly controlled to prevent interference with subsequent experiments [31]. The sample needs to select the appropriate translation text. For this experiment, 100 professional translators, 150 students, and 50 ordinary people were randomly interviewed by means of questionnaires. It investigates the translation fields commonly used by these people and the proportion of various types of sentences in translation and makes a statistic on the words or sentences they often translate.  Table 1 is a statistical table of translation samples.

It can be seen from the data in Table 1 that professional translators account for a large proportion of the translation of professional terms and professional acronyms. Ordinary people translate almost only everyday language. The proportion of student translation is relatively neutral.

#### 4.1.2. Correlation of Samples

In the sample translation experiment, the selection of samples will greatly affect the test results. Some data have little effect on the experimental results, but some data can change the experimental results. These extreme data are experimental and should be noted [32]. Correlation analysis is to solve the problem of improper selection of these sample data. Through the correlation analysis, the main features can be made clear, and it can be clearly seen which factors have a greater impact on the system. According to the data in Table 1, a total of 5 professional terms (options; internal combustion engine; quantumtheory; blackhole; squareroot), 3 acronyms (USA; ANN; AI), and 5 common sentences (Come on; See you; Here you are; Good luck; This way) were selected as the analysis data of this translation sample correlation test.  Table 2 is the correlation analysis table of translation samples.

From the data in Table 2, it can be seen that the 13 sample indicators are related to the translation system. Each indicator has a great influence on the results of the system, and considering that the dimension of the data used in this experiment is not high, all the above 13 samples are used as the sample data for evaluating the translation system.

#### 4.1.3. Validity of the Sample

In order to test whether the sample is valid for the translation system, this experiment is carried out by means of *k*-fold cross-validation. That is to divide all the data into *k* equal parts and run the experiment *k* times. In each run, one of them is selected as the test data, the other *k* − 1 as the test data, and the final test result is the average of the *k* test results [33]. Since the dimension of this experiment is not large, 4-fold cross-validation is selected. 400 sets of data are selected for the experiment, of which 80 sets of data are test groups, and the remaining 320 groups are exam groups. This method is applied to machine-assisted English translation systems and machine English translation systems, respectively.

The 4-fold cross-check results of the Artificial Intelligence-based machine-assisted English translation system and the machine-to-English translation system are shown in Table 3:

Through the analysis of the data in Table 3, the correct translation rate of the machine-assisted English translation system based on artificial intelligence is 96.0%, and the wrong translation rate is 4.0%. The correct translation rate of the machine English translation system is 84.0%, and the incorrect translation rate is 16.0%. Since the translation accuracy of the two models is high, a translation comparison test of the two models can be carried out.

### 4.2. Comparison Experiment between Machine-Assisted English Translation and Machine English Translation

In order to find a translation mode that can largely replace human translation, this experiment selects a machine-assisted English translation system based on artificial intelligence and a machine English translation system for multifaceted comparison. The Artificial Intelligence-based machine-assisted English translation system is based on translation memory. It learns to translate through convolutional neural networks and deep Boltzmann machines. Machine English translation is trained by an artificial neural network to match the translation. In the following experiments, the machine English translation will select Google Translate [34, 35], which has a better translation effect.

Because machine-assisted English translation has a good recognition effect on professional English, machine English translation has a poor translation effect on professional English. The experiment sets a matching degree. Match degree means the percentage of characters and formats in the field to the content of the translation memory. The experiment will test the translation quality and translation efficiency of the two translation modes under different matching degrees. The experimental matching degree is set to be less than 60%, 60%–80%, and greater than 80%, respectively.

#### 4.2.1. The Matching Degree Is Less Than 60%

In order to test two different translation models, the experiment will select the same text for translation. For the convenience of recording errors and types of errors, the experiment has compiled a list of common translation errors for reference. Common types of translation errors are shown in Table 4.

When the matching degree is set to less than 60%, the mistranslation distributions of the two translation models are shown in Figure 6:

It can be seen from the analysis in Figure 6 that when the matching rate is less than 60%, the types and numbers of translation errors in the Artificial Intelligence-based machine-assisted English translation system are similar to those in the machine-English translation system. Artificial Intelligence-based machine-assisted English translation systems start off with more mistakes than machine-to-English translation systems, but as the translation progresses, the machine learns to make the gap between the two gradually narrow. Mistranslation of terms and mistranslations of acronyms accounted for the largest proportion of errors in machine English translation. The error rate of machine-assisted translation is not very high in these two error types.

#### 4.2.2. The Matching Degree is 60%–80%

When the matching degree is set between 60% and 80%, the mistranslation distributions of the two translation models are shown in Figure 7.

It can be seen from the analysis in Figure 7 that when the matching rate is between 60% and 80%, the number of translation errors in the Artificial Intelligence-based machine-assisted English translation system is much less than that of the machine-English translation system. Moreover, the types of errors in machine-assisted English translation are more evenly distributed in terms of error types. Machine English translation has a high proportion of translation errors in professional English and acronyms. All in all, as the matching rate increases, so does the translation accuracy of the machine-assisted English translation. The translation efficiency and quality are much better than machine English translation.

#### 4.2.3. The Matching Degree Is Greater Than 80%

When the matching degree is set greater than 80%, the mistranslation distributions of the two translation models are shown in Figure 8.

From the analysis of Figure 8, it can be seen that when the matching rate is greater than 80%, the number of translation errors in the Artificial Intelligence-based machine-assisted English translation system is far less than that of the machine-English translation system. In terms of error types, the types of errors in machine-assisted English translation are mainly simple vocabulary errors. Machine English translation has a high proportion of translation errors in professional English and acronyms. When the matching rate is greater than 80%, the translation accuracy of machine-assisted English translation increases exponentially. The translation efficiency and quality are much better than machine English translation.

#### 4.2.4. Experimental Results

From the point of view of the matching rate, the experiment sets the matching rate of three gradients with a matching rate of less than 60%, between 60% and 80%, and greater than 80%. With the improvement of the matching rate of the experimental data, the error rate of the machine-assisted English translation system based on artificial intelligence is greatly reduced. In just 0.5 seconds, the number of errors dropped from 12 to 3. In addition, the proportion of errors in professional English and acronyms and other professional words has also dropped significantly. In contrast to machine English translation, the number of errors increases proportionally with the increase of time. The proportion of errors is mainly professional English and acronyms. However, when analyzing the two translation models in the face of simple vocabulary, the efficiency of machine English translation is slightly better than that of machine-assisted English translation, as shown in Figure 9. In summary, the advantages of machine English-assisted translation in terminology processing are illustrated. Machine English-assisted translation can improve translation and translation quality faster. However, in the face of pure and simple vocabulary, the translation efficiency and quality of machine English-assisted translation are slightly inferior.

## 5. Discussion

With the development of artificial intelligence technology, the combination of “Internet of Things+” and various fields has had a huge impact on social production, education, and life. Although machine English translation has a good translation efficiency, it often makes mistakes when dealing with terminology, repeated sentences, and complex sentences in large paragraphs. Therefore, artificial intelligence is applied to the translation field, using convolutional neural networks and deep learning techniques to model machine English-assisted translation. It builds a translation memory knowledge base through the system's self-learning ability. This enables the machine English-assisted translation system to take advantage of processing terms and complex sentences and maximize the help of human beings to achieve text translation. However, when conducting machine translation comparison experiments, no advanced data preparation and result estimation were made.

## 6. Conclusions

By comparing Artificial Intelligence-based machine English-assisted translation with ordinary machine English translation (Google Translate), the following conclusions are drawn: (1) According to the statistics in the error analysis, Artificial Intelligence-based machine-English-assisted translation terms have few translation errors. 7 errors in machine English translation are caused by term mistranslation. Terminology mistranslations account for about 30% of all translation errors made by Google Translate. Artificial Intelligence-based machine English assistance is mostly lexical errors. Machine English translation is mainly for lexical errors and syntactic errors. And when the matching rate is as high as 80% or more, there are very few errors in the machine English assistance based on artificial intelligence. (2) When faced with short and simple sentences, the efficiency of machine English translation is higher. Artificial Intelligence-based machine English assistance is more efficient when translating long complex sentences or acronyms. In summary, the advantages of machine English-assisted translation in terminology processing are illustrated. Machine English-assisted translation can improve translation and translation quality faster.

## Figures and Tables

**Figure 1:** BP neural network structure diagram.

**Figure 2:** Convolutional neural network structure diagram.

**Figure 3:** Subsampling layer sampling diagram.

**Figure 4:** Structure diagram of deep belief network.

**Figure 5:** Structure diagram of deep Bozeman machine.

**Figure 6:** Mistranslation distribution with a matching rate less than 60%. (a) Error type distribution map. (b) Distribution map of the number of errors.

**Figure 7:** Distribution of mistranslations with matching rates between 60% and 80%. (a) Error type distribution map. (b) Distribution map of the number of errors.

**Figure 8:** Mistranslation distribution when the matching rate is greater than 80%. (a) Error type distribution map. (b) Distribution map of the number of errors.

**Figure 9:** Mistranslation diagram for translating simple words. (a) Error number distribution map. (b) Translation efficiency distribution map.

**Table 1:** Translation sample statistics.

Phrase classification	Professional translator (%)	Student (%)	Ordinary people (%)
Terminology	60	30	5
Acronym	20	20	5
Daily languages	15	40	80
Other	5	10	10

**Table 2:** Translation sample correlation analysis table.

Number ofsample groups	Translation phrase	Relevance
1	Options	0.0613
2	Internal combustion engine	0.0994
3	Quantumtheory	0.0535
4	Blackhole	0.1274
5	Squareroot	0.0153
6	USA	0.0834
7	ANN	0.0595
8	AI	0.0714
9	Come on	0.1075
10	See you	0.0354
11	Here you are	0.1183
12	Good luck	0.0244
13	This way	0.0964

**Table 3:** English translation cross-check table.

Translation phrase	Correct translation rate of assisted translation (%)	Wrong translation rate of assisted translation (%)	Correct translation rate of machine translation (%)	Wrong translation rate of machine translation (%)
Terminology	95.3	4.7	75.3	24.7
Acronym	98.8	1.2	74.5	25.5
Daily languages	94.4	5.6	93.5	6.5
Other	95.6	4.4	92.7	7.3
Average	96.0	4.0	84.0	16.0

**Table 4:** Table of common translation error types.

Serial number	Error type
1	Lexical error
2	Add word
3	Term mistranslation
4	Mistranslation of acronyms
5	Capitalization error
6	Omit
7	Conjunction mistranslation
8	Part of speech error
9	Punctuation error

## Data Availability

The data that support the findings of this study are available from the corresponding author upon reasonable request.
